# Urban Management in the Dynamic Relationship between the Occurrence of Environmental Pollution Accidents and Economic Development in China

**DOI:** 10.1155/2022/3751028

**Published:** 2022-08-28

**Authors:** Xuwen Cong, Huaixing Wang, Jingmei Huang

**Affiliations:** ^1^School of Administration, Changchun University, Changchun, Jilin 130022, China; ^2^School of Politics and Law, Northeast Normal University, Changchun, Jilin 130024, China

## Abstract

After the reform and opening up, China has developed into a world factory due to the bias of Chinese policies, the need for urban development, and the limitations of science and technology. As a world factory, on the one hand, it expanded the scale of China's economy, raised the level of science and technology, and improved the standard of people's daily life. On the other hand, China's technology level was backward at the beginning of the reform and opening-up period, and the world countries in a competitive relationship could not give China a high-end technology level. Most of the developed countries only transferred their rough industries to China, which led to the “three highs and one low” pattern of China's economic development. The efficiency of resource utilization is very low, which not only wastes resources but also causes great deterioration of the environment. Based on China's environmental development problems, this article summarizes and analyses the relationship between economic development and environmental pollution through the perspective of EKC curve research. Then, using the data of economic growth target published by government work report of 230 prefecture-level cities from 2004 to 2014 collected by hand, the constraint of economic growth target is described from three dimensions. In particular, the study of economic growth target constraints is extended in terms of the portrayal of the characteristics of soft and hard constraints of economic growth targets. Finally, combining with the normative research method, feasible countermeasures are proposed for developed cities as well as less developed cities, providing new insights for the coordinated development of the urban environment and economy in China.

## 1. Introduction

Since the twenty-first century, excessive energy consumption has put a certain burden on the urban environment, such as excessive carbon emissions, air pollution, and a series of other ecological problems [1]. At present, the development and utilization of oil, natural gas, and coal in China's cities are on the right track, and the formation and operation of an industrial system based on the energy and chemical industry has been realized [2].

The relationship between the environment and the economy was further demonstrated [3]. Since then, several researchers have also verified the existence of EKC curves [4–6]. However, many scholars have also found that EKC curves are not universal [7]. Haseeb [8] studied the relationship between environment and economy using Malaysian national data and found that economic growth does not necessarily improve the environment.

Domestic scholars have also conducted numerous studies. Xu et al. [9] conducted an EKC validation on the data of Liaoning Province from 1985 to 2004. Sun et al. analysed the relationship between greenhouse gases and the economy in China, which is consistent with the EKC and analysed the inflection point of the EKC [10]. They argue that if GHG emissions are not reduced in the future, future environmental pressures will exceed China's environmental carrying capacity. Literature [11] found that the relationship between the three industrial wastes and the economy in Qingdao is only partially consistent with EKC. Literature [12] used data from 1996 to 2009 to construct panel data, and it was concluded that technological progress led to negative environmental development instead.

This article takes the growth target data mentioned in the government work report economy of 230 prefecture-level cities in China from 2004 to 2014 as the research sample. It focuses on the study of the impact of economic growth target constraints on local environmental pollution and proposes different feasible countermeasures through the analysis of the economic development status of different cities.

The innovative points of this article are as follows:

1. Based on the perspective of economic growth target setting, it provides a new perspective for the study of urban environmental pollution.
2. It brings enlightenment to the policies of government performance evaluation and economic growth target management.
3. It provides a new idea for solving the problem of urban environmental pollution management.

The rest of the article is organized as follows: Section 2 details the state of the art, Section 3 describes the methodology, Section 4 provides result analysis and discussion, and Section 5 concludes the article.

## 2. State of the Art

Research on the relationship between economic development and environmental pollution has focused on the environmental Kuznets curve (EKC) (See Figure 1).

The theory of EKC has been further enriched and improved as the theoretical discussion on environmental pollution and economic development continues to intensify.

According to different analytical perspectives, the theoretical studies on environmental pollution and economic growth are divided into two main categories. The first category adds environmental constraints to the neoclassical growth model and examines the changes in economic growth paths after adding environmental constraints. The second category adds environmental constraints to the endogenous growth model and explores the issue of sustainable economic growth.

The neoclassical growth model is a model of economic growth proposed by [13] and others. It continues the assumptions of neoclassical economics. Under this assumption, it is concluded that the economic growth rate is equal to the population growth rate when the variable of capital per capita is zero and the level of technology is constant. Literature [14] developed a two-sector model (production sector and pollution reduction sector). The model analysis suggests that to keep the economy growing at a balanced rate, it is necessary to reduce the level of consumption and increase the capital stock by controlling investment appropriately. Literature [15] found that pollution is a by-product of the production process, but the presence of pollution does not affect the conclusions of the study. The long-run growth rate of the economy does not change, but it reduces the capital-intensive production process. Literature [16] in his article constructs a general equilibrium model with only two countries (South and North), and the key variables are property rights and institutions. In this model, there are clear property rights of the environment in the North, whereas the South has no property rights in the environment, so adjusting prices through international trade will not lead to a decrease in environmental pollution, but rather to a deterioration of the environment on both sides. Literature [17] used a generational overlap model to investigate the relationship between environmental investment and environmental quality issues. In this model, the utility from environmental investment is low and the utility from consumption is high in the early stage of economic development, and people are more willing to consume. In the later stages of economic development, the utility from consumption is lower than the utility from the environment. Literature [18] extended the Solow model to form the “Green Solow model.” Their study shows that in the long run, the adoption of severe pollution reduction policies is not effective in promoting economic growth, while technological advances in product production and cleaner pollution will largely improve environmental conditions.

The endogenous growth model breaks through the original hypothesis of the neoclassical growth model based on the neoclassical growth theory and endogenously generates some variables. It mainly includes the knowledge spillover model of Romer (1986); the “AK” model of Barro (1990) and Robelo (1991); and the human capital externality model of Lucas (1988). Based on Romer's model, it can be found that government subsidies to environmental departments and certain environmental taxes increase in a balanced way [19]. The model shows that when per capita income is low, the positive utility of a unit of consumption is much greater than the negative utility of a unit of pollution to consumers. The total utility of using high pollution industries is positive, so the economic development will bring down the environmental level. When income increases to a certain level, the total utility of high pollution industries will change from positive to negative due to the law of diminishing marginal utility, people will reduce consumption in exchange for the rise of environmental quality, and enterprise production will be based on low pollution production technology. Literature [20] added new elements to Lucas's human capital model. They argue that environmental pollution reduces learning and explores how economies grow in the long run when society as a whole prefers a “good” environment. They argue that adopting a high standard of environmental measures in a short time frame can reduce output and inhibit economic development. But over a longer period of time, it boosts productivity and accelerates economic growth. Literature [21] developed a “kindergarten sustainability rule” model. The model shows that when economic income is low, there is a big difference in the level of environmental pollution in different regions. When the economic income increases, the environmental pollution levels of different regions will be close to the same, which leads to the idea that the environmental pollution levels of developed and underdeveloped regions will eventually converge. At the same time, it is analysed that to achieve sustainable development, it is not necessary to rely on increasing income; instead, it is also important to find effective ways to improve the return on environmental investment or to invent completely pollution-free technology.

## 3. Methodology

In the context of economic globalization, international environmental problems such as greenhouse effect, acid rain, and ozone hole have become potential threats to human survival and development. As the largest developing country, China is experiencing rapid economic development while the pressure of environmental pollution is increasing day by day. The dead fish in Baiyangdian in Hebei; the massive outbreak of cyanobacteria in lakes such as Taihu Lake, Chaohu Lake, and Dianchi Lake; the crude oil spill in Xingang, Dalian; and the growing haze in cities are all signs of deteriorating ecological conditions that pollutant emissions are exceeding environmental carrying capacity.

The World Environmental Performance Index (EPI) report systematically assesses the environmental performance of economies based on changes in scores for 24 specific assessment indicators in 10 policy areas, which include air pollution, water resources, water and sanitation, biodiversity and habitat, forests, fisheries, climate and energy, heavy metals, agriculture, and air quality across countries and regions.

China's overall environmental performance score has always been at the bottom of the EPI rankings.  Figure 2 shows how China's ranking has changed over the years in the EPI assessment. It can be seen that among the participating countries, China's environmental performance ranking is not good. In 2012, China's environmental performance ranking was the lowest ever, ranking in the bottom 16. China's environmental performance assessment began to improve after a period of decline between 2006 and 2018. On balance, China's environmental performance is now on a steady upward trend compared to 2006. Specifically, the EPI scores of specific indicators in China in 2018 and 2007 were used for comparative analysis. The results are shown in Table 1. Over the past 10 years, China's overall environmental performance has increased steadily, from a score of 46.36 and a ranking of 136 in 2007 to a score of 51.85 and a ranking of 120 in 2018, with China excelling in the areas of fisheries (ranked 17), climate and energy (ranked 20), and water and sanitation (ranked 47), above the other areas. However, it is easy to see from the table that problems are more prominent in the area of air quality. In particular, the average and excellence rate of PM2.5 exposure are very low, resulting in a score of 15.5 in the air quality domain and a ranking of 177. The lagging air quality domain seriously affects the overall score of China's environmental performance.

### 3.1. Water Pollution Status

In addition to the uneven distribution and relative scarcity of water resources in China, the pollution problem is also prominent. The main pollution indicators of water resources in China include total phosphorus, chemical oxygen demand, and permanganate index. According to the 2017 China Ecological Environment Bulletin, 67.9% of the surface water bodies in China are good (Class I–III), 23.8% belong to Classes IV and V, and 8.3% are poor (Class V). This means that more than 30% of the surface water bodies in China are still polluted. That is to say, there are still more than 30% of water bodies that do not meet the standard. In the lake (reservoir) water bodies, as can be seen from Figure 3, 112 important lakes (reservoirs), I–III water quality of the number of lakes (reservoirs) is 70, accounting for 62.5%. The number of IV and V is 30, accounting for 26.8%. Poor V for 12, accounting for 10.7%. The public is aware of the heavy, moderate, and light pollution levels in the Dianchi, Chaohu, and Taihu lakes.

Table 2 reflects the discharge of wastewater in China from 2011 to 2015. From the table, it can be seen that the total wastewater discharge in China has increased year by year. As for the main pollution indexes, the chemical oxygen demand and ammonia nitrogen emissions reached the maximum in 2011, with 2622.9 million tons and 272.7 million tons, respectively. After 2011, they both show a slow decline year by year. In 2015, the discharge of chemical oxygen demand and ammonia nitrogen in industrial wastewater were at the lowest level in all years. From the above analysis, we can see that although the water pollution in China is still serious and not optimistic, it is in a state of slow improvement.

Figure 4 reflects the changes in total wastewater discharge in each region. In 2011, the wastewater discharges in the eastern, central, and western regions were 35.313 billion tons, 17.713 billion tons, and 12.893 billion tons, respectively. In 2015, the volume of wastewater discharged in different places slightly increased to 38.62 billion tons, 19.86 billion tons, and 15.052 billion tons, respectively. In 2016, China's wastewater discharges declined for the first time during the sample period, falling to 37.702 and 18.121 billion tons in the eastern and central regions, respectively. Although emissions in the western region still increased to 15.287 billion tons, the total wastewater discharge in China decreased to 71.110 billion tons from 73.532 billion tons in 2015. To a certain extent, the reduction of wastewater emissions in the eastern and central regions is beneficial to the overall reduction of wastewater emissions in China. In addition, during the sample period of 2011–2016, the wastewater emissions of each region to the total national wastewater emissions always show the phenomenon of east > central > west. In particular, the eastern region accounts for about 53% of the wastewater discharge, which is always much higher than that of the central and western regions. Taking 2016 as an example, the proportion of wastewater in the eastern central, and western regions is 53.02%, 25.48%, and 21.50%, respectively.

Table 3 further depicts the emission status of typical pollutants by region in 2016. Take chemical oxygen demand emissions as an example, the eastern, central, and western regions accounted for 39.92%, 31.90%, and 28.18%, respectively. As for some heavy metal emission indicators, such as lead, mercury, cadmium, arsenic, and other heavy metal elements, the phenomenon of central > western > eastern shows. Taking lead emission in each region as an example, the central, western, and eastern regions account for 52.44%, 33.84%, and 13.71% of the emission, respectively. It can be seen that there are large differences in the total amount of wastewater discharge and the main pollutants in wastewater in each region of China.

### 3.2. Air Pollution Status

In the 2018 Global Environmental Performance Assessment report, China's lag in the area of air quality seriously affects its overall environmental performance score, with the extent and harm of air pollution becoming increasingly serious. Only 99 of the 338 prefecture-level cities and above, or 29.3% of the sample prefecture-level cities, achieved ambient air quality standards (AQI index in the 0–100 range). The number of cities with AQI greater than 100 exceeded the standard was 239, accounting for 70.7%.

Air pollution in China can be broadly classified as follows: (1) A sharp increase in emissions of sulphur-containing pollutants due to the increasing consumption of coal resources, which further causes the expansion of the scope of acid rain; (2) an increasing number of motor vehicles, resulting in a sharp increase in tailpipe emissions of pollutants such as nitrogen oxide emissions; and (3) industrial development such as thermal power plants and industrial boilers lead to smoke and dust emissions.

Figure 5 reflects the emissions of major air pollutants in China from 2011 to 2016; in general, the emissions of sulphur dioxide, nitrogen oxides, and smoke (dust) have decreased, from 22.1791 million tons, 240.427 million tons, and 12.7883 million tons in 2011 to 110.286 million tons, 13.9431 million tons, and 10.166 million tons in 2016, respectively. The reduction was about 50.27%, 42.01%, and 20.97%, respectively. Smoke (dust) emissions increased from 2013 to 2014. After 2014, smoke (dust) emissions started to decrease year by year. Overall, the air pollution situation in China is relatively serious. With the vigorous implementation of corresponding national policies, some progress has been made in reducing emissions, pollutant emissions have been reduced, and environmental quality has improved slightly. However, the work on environmental protection, especially air quality, is still arduous.

The emissions of air pollutants show more significant regional differences as wastewater. As shown in Table 4, the emissions of sulphur dioxide and nitrogen oxides showed a decreasing trend year by year during 2011–2016. Smoke (dust) emissions increased in 2013 and 2014 and then also showed a decreasing trend. During the sample period, the proportion of the three types of air pollutant emissions in the eastern, central, and western regions remained relatively stable. The eastern region has a larger share in the emissions of all three pollutants. In particular, the proportion of nitrogen oxide emissions and smoke (dust) emissions exceeded 40%. In terms of NOx emissions, in 2016, the eastern, central, and western regions accounted for 597.86 million tons, 418.34 million tons, and 415 million tons, respectively, accounting for 42.00%, 29.12%, and 28.88% of the national NOx emissions. Compared with 113.27 million tons, 737.03 million tons, and 690.87 million tons in 2011, they are reduced by 41.50%, 43.97%, and 40.65%, respectively. In terms of smoke (dust) emissions, in 2016, for example, the eastern, central, and western regions emitted 428.92 million tons, 309.15 million tons, and 309.5 million tons, respectively, accounting for 41.22%, 29.37%, and 29.41% of the country, compared with 457.02 million tons, 458.8 million tons, and 399.91 million tons in 2011, achieving 6.32% and 33.52%, respectively. Compared with those data in 2011, the proportion of emission reduction was 6.32%, 33.52%, and 23.33% respectively.

In terms of sulphur dioxide emissions, compared with the emissions of 804.29 million tons, 629.23 million tons, and 821.28 million tons in the eastern, central, and western regions in 2011, their emissions decreased to 413.11 million tons, 294.02 million tons, and 432.64 million tons, respectively, in 2016, a reduction of 49.39%, 54.34%, and 48.04%, respectively. Of particular concern is that the central region in terms of sulphur dioxide emissions, from 27.82% in 2011 to 25.54% in 2016, achieving the lowest in all years. While the eastern and western regions, relatively speaking, although compared to the 2011 emissions on the emissions achieved 49.39% and 48.04% reduction in emissions, they still occupy a large proportion of the regional share of sulphur dioxide emissions, accounting for 36.34% and 38.11%, respectively. Overall, although the emissions of air pollutants have decreased in all regions, the eastern region still has a larger share in the emissions of the three types of air pollutants and has a more significant impact on air quality than other regions.

### 3.3. Current Status of Economic Growth Target Setting

The central government has gradually turned the driving force of economic development to a new growth point driven by innovation and turned the mode of economic development to quality and efficiency intensive growth so as to achieve sustainable and stable economic growth. Although the central government is changing its setting of economic growth goals to adopt more coordinated and sustainable methods such as expected goals, the change of this concept has not been well implemented in lower-level governments.

At this stage, the explicit mode of governance targeting economic growth and the invisible mode of governance mainly based on person tenure and cross-location exchange are still the main modes of governance of local officials by the central government. The “cascading” is reflected at the lower levels of government, with a tendency to increase the value of economic growth target set by higher levels of government (see Table 5). Table 5 shows that the average economic growth target set by local governments at the municipal level is 1.05%–2.83% higher than the average economic growth target set by the provinces where they are located, and the excess is 11%–27% of the economic growth target set by the provinces where they are located. Similarly, the average economic growth target set by local governments at the municipal level is 2.8%–5.3% higher than those set by the state. In particular, after 2005, Table 5 shows that the average difference between municipal and provincial targets jumped to 2.543% in 2006 compared to 1.984% in 2005. Therefore, this article considers 2006 as a critical point in time. Further, since the arithmetic mean of cities or provinces is used for comparison, we cannot exclude that there are extreme values in individual cities or provinces that affect the mean value. For this reason, this article presents a grouping of the differences. As shown in Figure 6, the difference between the economic growth target of prefecture-level cities and that of their provinces is greater than 2% in more than 50% of the cities and only 2.77% of the prefecture-level cities have an economic growth target smaller than that of their provinces. The difference between the municipalities and the country is more obvious, with more than half of the municipalities having a growth target greater than 4%. And less than the national target value occurs only 22 times, accounting for 0.87%. This shows that most of the provinces and cities in China have increased their economic growth targets at this stage, and the lower the level of government, the more obvious the phenomenon of “cascading increases” is.

Although the government has changed the terminology of setting economic growth targets from “ensure” to “expect,” the weakening of the hard constraint characteristics of the central government's economic growth target has not caused a big change at the provincial and municipal levels.

From Table 6, some local governments still adopt the terms with more obvious hard constraint characteristics to set economic growth targets. Between 2010 and 2016, about 80% of the sample size of prefectures adopted the language of hard constraints to set economic growth targets. In 2010, only 20 prefectures out of 230 prefectures adopted the soft constraint language of “leaving room” to set economic growth targets, while as many as 210 prefectures adopted the language of hard constraints. In 2016, as many as 144 prefectures, accounting for 62.61%, still adopted hard constraint terms. In general, among the 230 prefectures, although the number of prefectures adopting the soft constraint terms of “left and right” has gradually increased in recent years, the total number is still low, accounting for less than 20%. Among the prefectures in the sample, most of them still adopt the hard constraint terms such as “ensure,” “above,” and “achieve” as the terms. The majority of the prefectures in the sample still use hard and binding terms such as “ensure,” “above,” and “achieve” as their economic growth targets.

It can be seen that the municipalities can exceed their growth targets. However, in recent years since 2011, there have been instances where the growth targets were set too high to be achieved. In terms of the regional distribution of the overachievement, the eastern provinces and cities have done better than the central and western provinces and cities. Although economic growth targets as a kind of expectation may be disturbed by many unpredictable factors in actual accomplishment, the targets should have their own flexibility and scientificity. For those regions that failed to achieve their targets, the reason is that their economic growth targets deviated from the potential growth rates in line with their regional factor endowments.

As shown in Table 7, it can be found that the target economic growth is mainly concentrated in the range of 10%–15%, accounting for 78.7% of the total, while those exceeding 15% account for 12.61%. The actual achievement is also concentrated in the range of 10%–15%, accounting for 60.79%, while those exceeding 15% account for 23.56%. In terms of the difference between the completion value and the target value, the sample size of 0–2% is the largest at 908, accounting for 35.89%, but the sample size in the interval of −10% −0 also reaches 33.52%, while the failure to achieve its target value accounts for 34.19%. In other words, more than one-third of the sample failed to achieve the growth target. Overall, the actual overachievement of economic growth targets is not optimistic.

## 4. Result Analysis and Discussion

### 4.1. Build a Sustainable Development System of the City

For a region to achieve sustainable development, it must first recognize reality and have a very clear understanding of its own development. Both cities and villages in China do not have a full understanding of themselves. The first is the lack of environmental pollution statistics. From the environmental statistics of different cities, there are more missing data of environmental pollutant emission data in each provincial capital city, and many pollution emission data are not counted. Most of the data used by scholars rely on other data for estimation, such as carbon dioxide, some domestic pollutant emissions, etc. The lack of data in cities of lower levels is even more serious. The second is the lack of positive environmental statistics. For the environment, while we pollute the environment, we are also carrying out positive activities such as energy saving and emission reduction, afforestation, and increased greening. Therefore, from the perspective of environmental statistics, we should construct a comprehensive level of indicators to measure the level of sustainability of a city. Not only the air quality of an area should be considered but also the water environment, air environment, noise environment, human environment, and other factors.

### 4.2. Increase the Support for Scientific Research and Technology Promotion

Technological progress can reduce the cost of pollution control, making the same environmental control funds have a higher utilization rate. Technological progress can reduce the environmental input in production activities, making less environmental input to get the same economic output. Technological progress can reduce the environmental pollution output of people's lives and help achieve low-carbon consumption, such as reducing automobile emissions and increasing the rate of waste disposal. The second is to increase support for the promotion of technology, the emergence of new technology is often the need to promote. And enterprises for the replacement time is often a long cycle, making the utilization of new technologies low. Therefore, we should support enterprises through policy and funding and improve the consciousness and initiative of enterprises.

### 4.3. Raising People's Awareness of Environmental Protection

Raising the awareness of environmental protection among all people is the only way to reduce environmental pollution in many aspects, such as production aspect, distribution aspect, exchange aspect, consumption aspect, and use aspect. Carry out in-depth education on environmental protection. Make the concept of environmental protection deeply rooted in people's hearts and make environmental protection behaviour instinctive. Only education can make people realize the seriousness of environmental problems, develop their environmental awareness, and acquire skills and methods to protect the environment.

Foster environmental groups and organizations. The environment is a “public good” and people often have a “free-rider” mentality, which makes it difficult to increase their motivation to protect the environment. In the face of this dilemma, the government should strongly support private environmental groups and organizations and standardize and institutionalize these organizations and their activities. At the same time, to increase people's participation in environmental activities, the government should work with environmental groups to expand the scope of environmental policy responses through these groups as well as increase their number and influence.

### 4.4. Population Diversion

The high level of development in developed cities has attracted a large number of foreigners. The continuous influx of foreign population brings prosperity to the city's economy, but at the same time brings huge bearing pressure to the city. There is an upper limit to the environmental carrying capacity of a city. As the resident and mobile populations in developed cities continue to rise, the environmental carrying capacity of cities is beginning to struggle to withstand such a large population and various urban environmental problems are emerging. Therefore, developed cities should first optimize the population structure in a planned way to achieve a positive interaction between population and industry. Second, they should support the development of neighbouring cities, which, on the one hand, promotes the overall development of China and, on the other hand, shares their own pressure. Finally, they should give up some non-advantaged industries and transfer these industries to places where they can tap the potential to achieve the purpose of population diversion.

### 4.5. Reduce Environmental Pollution from Domestic Waste

The environmental pollution caused by domestic pollutants in cities can no longer be ignored. This problem is more prominent in developed cities. First, developed cities have a higher level of development, and the government and enterprises pay much attention to environmental pollution caused by production activities but ignore the environmental pollution caused by domestic pollutants. Second, the population of developed cities is more attractive than less developed cities. Therefore, developed cities have a large population and produce far more domestic pollutants than less developed cities. So developed cities should, on the one hand, increase technological innovation in clean living pollution, reduce the rate of living pollutants generated, promote the reuse of living pollutants, and improve the rate of living pollutants treatment. On the other hand, they should improve the level of environmental infrastructure, formulate relevant policies, and implement relevant measures to reduce the impact of living pollutants on the environment.

### 4.6. Learn from the Development Experience of Developed Cities and Combine Their Own Advantages to Get Out of Their Own Way

The problem of the unreasonable and imperfect economic structure of less developed cities is very prominent. First, the single industrial structure and imbalance are common phenomena. Once the industry loses its power, the development of the city will stagnate; the industrial imbalance causes heavy industrialization of the industrial structure, which leads to high consumption of resources and serious pollution to the environment. The main problems of less developed cities are overcapacity and under demand.

The problem of overcapacity is a problem that has arisen in many cities at this stage, especially in less developed cities. The main reason is because of the consumption upgrade, which has led to a decline in demand for certain industries, which in turn has created the problem of overcapacity. As the industries in less developed cities are more homogeneous, the problem of overcapacity is further magnified. Therefore, the first thing for less developed cities is to improve the industrial structure of the cities. By vigorously promoting independent innovation, they can find the fulcrum for improving the industrial structure, cultivating new strategic industries, and driving the development of other industries. The second is to let the surplus industries “go out.” Through industrial transfer, the surplus industries will be transferred to other countries with lower development levels. The third is to purposefully eliminate industries with no development potential and replace them with new industries. The fourth is to merge and reorganize industries that still have development potential to improve the competitiveness of the industry.

Insufficient domestic demand is also one of the main problems in less developed cities and leads to insufficient development momentum of cities. In less developed cities, the economic level is backward, the purchasing power of urban residents is insufficient, the traditional consumption concept is deep-rooted, the social security system is not perfect, the income level of residents is low, and so on, which leads to the lack of domestic demand in cities. Therefore, the government should formulate relevant policies and take relevant measures to expand domestic demand. For example, the government should implement a proactive fiscal policy and use relevant economic tools to stimulate consumption, create consumption hotspots, improve residents' consumption environment, and change their consumption concepts.

## 5. Conclusion

In the past, China's economic growth was too brutal, similar to the early capital development, because of the “pollution sanctuary hypothesis” and technological limitations. However, such economic growth is not suitable for the current era, and one of the most important points is that it ignores the deterioration of the environment. Environmental degradation has started to affect people's normal life and people's life and health. Therefore, in this article, the relationship between economic development and environmental pollution is studied by applying the environmental Kuznets curve theory. The relationship between economic growth targets and environmental pollution is described and analysed in terms of environmental quality, water pollution, and air pollution. The data related to economic growth targets in 230 city government work reports were collected. The economic growth target constraints are portrayed in three dimensions: cascading, constraint characteristics, and overachievement. Finally, different countermeasure suggestions are proposed by targeting cities with different economic development status. Due to the different geographical locations and natural environmental conditions of each city, the structure and development methods of urban economic development are different. Subsequent studies will further add the abovementioned and other factors to the classification of cities and improve the selection of urbanization indicators to make this study more enriched and provide a solid theoretical foundation and basis for the sustainable development of cities.

## Figures and Tables

**Figure 1:** Environmental Kuznets curve.

**Figure 2:** Change in China's EPI ranking.

**Figure 3:** Analysis of water quality categories of lakes (reservoirs) in China in 2017.

**Figure 4:** Total wastewater discharge by region, 2011–2016 (billion tons).

**Figure 5:** Major air pollutant emissions (unit: million tons).

**Figure 6:** Gap in economic growth target setting between city and province and city and country, 2004–2014.

**Table 1:** China's EPI indicator assessment scores (selected indicators).

EPI	Target	Policy areas	Indicators	In 2018		In 2007	
				Ranking	Score	Ranking	Score
Environmental performance index	Population	Overall	Overall	120	51.85	136	46.36
	Environmental health	Overall	Overall	167	32.83	175	23.36
		Air quality	Overall	177	15.5	177	8.56
			Household solid fuels	110	26.96	118	15.18
			Average PM2.5 exposure	177	2.16	178	1.23
			Exceedance rate of PM2.5	177	13.55	178	7.07
		Water and sanitation	Overall	47	69.35	77	53.94
		Heavy metals	Lead exposure	130	39.13	137	32.27
	Ecosystem vitality	Overall	Overall	39	64.53	44	61.69
		Biodiversity and habitat	Overall	100	73.68	81	75.54
		Forests	Tree cover loss	72	23	63	32.67
		Fisheries	Overall	17	71.52	46	65.61
		Climate and energy	Overall	20	69.73	67	52.82
		Air pollution	Total	62	58.19	33	71.95
			SO_2_ emissions	65	61.23	35	76.57
			NO_x_ emissions	65	55.16	40	67.33
		Water resources	Wastewater treatment	66	81.31	66	81.43
		Agriculture	Sustainable nitrogen management	61	35.75	61	35.87

**Table 2:** 2011–2015 national wastewater discharge.

Year	Wastewater emissions (billion tons)	Industrial	Domestic	Chemical oxygen demand emissions (million tons)	Industrial	Living	Ammonia nitrogen emissions (million tons)	Industrial	Domestic
2011	671.5	243.2	440.2	2622.9	367.1	951.1	272.7	29.33	160
2012	697.1	233.9	475	2546.7	350.8	925.1	265.9	27.63	156.9
2013	707.7	222.1	497.4	2475.7	331.8	902.1	258	25.83	153.7
2014	728.5	217.6	522.6	2417.6	323.7	876.7	250.8	24.43	150.5
2015	747.6	211.8	547.5	2346.5	305.8	859.2	242.2	22.93	146.4

**Table 3:** Emissions of major pollutants in wastewater in 2016.

Area	Chemical oxygen demand (million tons)	Ammonia nitrogen (million tons)	Total nitrogen (million tons)	Total phosphorus (million tons)	Petroleum (ton)	Volatile phenols (tons)	Lead (kg)	Mercury (kg)	Cadmium (kg)	Arsenic (kg)
National	1046.53	141.78	212.11	13.94	8838.7	381.2	52930.5	613	11219.4	41946.7

Eastern region	417.75	63.45	98.66	6.25	3207.1	81	7257.6	167.6	844.2	1783.6

Central region	333.86	43.05	63.28	3.95	3028.8	265.5	27759.4	308.7	7003.4	22813.8

Western region	294.93	35.28	50.2	3.74	2602.5	34.7	17913.5	136.6	3371.8	17349.5

Proportion in the eastern region (%)	39.92	44.75	46.51	44.84	36.28	21.25	13.71	27.34	7.52	4.25

Proportion in the central region (%)	31.90	30.36	29.83	28.34	34.27	69.65	52.44	50.36	62.42	54.39

Proportion in the western region (%)	28.18	24.88	23.67	26.83	29.44	9.10	33.84	22.28	30.05	41.36

**Table 4:** Air pollutant emissions by region (unit: million tons).

Year	SO_2_ emissions				NO_x_ emissions				Smoke (dust) emissions			
	National	East	Central	West	National	East	Central	West	National	East	Central	West
2011	2329.01	804.29	629.23	821.28	2515.37	113.27	737.03	690.87	1389.93	457.02	458.8	399.91
2012	2228.73	764.07	597.3	793.16	2448.86	973.52	709.49	691.65	1346.87	431.32	426.75	414.6
2013	2155.02	728.98	580.27	771.57	2338.4	907.44	679.32	677.5	1389.24	448.23	432.67	434.14
2014	2085.52	697.14	560.87	753.3	2189.1	844.6	637.51	632.79	1851.85	657.2	589.58	530.87
2015	1970.22	657.51	536.21	702.29	1962.12	755.16	568.77	563.99	1649.11	574.63	543.74	56.54
2016	1213.96	413.11	294.02	432.64	1505.41	597.86	418.34	415	1121.76	428.92	309.15	309.5

**Table 5:** Comparison of average values of provincial and municipal economic growth targets, 2004–2014.

Year	Municipal target	Provincial target	Difference between city and provincial targets	Difference between municipal and national targets	Municipal actual	Difference between city actual and provincial actual targets
2004	11.553	9.554	1.998	4.553	14.063	2.511
2005	12.049	10.065	1.984	4.049	13.855	1.806
2006	12.643	10.100	2.543	4.643	14.199	1.556
2007	12.929	10.157	2.772	4.929	15.024	2.095
2008	13.243	10.583	2.661	5.243	13.188	−0.055
2009	11.560	9.885	1.675	3.560	12.651	1.091
2010	12.316	10.054	2.261	4.316	14.410	2.094
2011	13.306	10.478	2.828	3.006	13.158	−0.148
2012	12.778	10.513	2.265	5.278	11.532	−1.247
2013	11.641	10.063	1.577	4.141	9.746	−1.894
2014	10.296	9.248	1.048	2.796	8.523	−1.773

**Table 6:** Statistics of economic growth target terms in prefecture-level municipal government work reports.

Year	National target (%)	City exceeds national target	Use “around”	Use “interval”	Use “ensure,” “above,” etc.	Use “achieve” etc.
2010	8	222	20	0	53	157
2011	8	228	24	0	56	150
2012	7.5	230	27	0	54	149
2013	7.5	228	42	0	51	137
2014	7.5	222	67	0	39	124
2015	7	182	65	1	31	133
2016	6.5–7	197	62	24	35	109

**Table 7:** Statistics of a high and low grouping of target overachievement in prefecture-level cities.

Variable	Economic growth target		Actual completed value		Variable	Difference between actual completion and target values	
Group (%)	Number of times	Percentage	Number of times	Percentage	Group	Group	Percentage
−5–0	0	0	3	0.12	Less than −10	17	0.67
0–5	1	0.04	51	2.02	−10–0	848	33.52
5–10	219	8.66	342	13.52	0–2	908	35.89
10–15	1991	78.70	1538	60.79	2–4	556	21.98
15–20	274	10.83	549	21.7	4–6	152	6.01
20–25	42	1.66	42	1.66	6–8	30	1.19
25–30	3	0.12	4	0.16	8–10	11	0.43
More than 30	0	0	1	0.04	More than or equal to 10	8	0.32
Total	2530	100	2530	100	Total	2530	100

## Data Availability

The labeled dataset that supports the findings of this study is available from the corresponding author upon request.
